# An Intelligent Recommendation Model for Health Culture Based on Short Video Content Analysis in the Mobile Internet Environment

**DOI:** 10.1155/2022/6009974

**Published:** 2022-09-16

**Authors:** Miao Ma, Xijing Zhang

**Affiliations:** ^1^Chengdu University of Technology, Chengdu 610059, China; ^2^Xijing University, Xian 710123, China

## Abstract

The heart and soul of the Chinese people and the greatest cultural soft power of contemporary China are excellent Chinese healthy cultural environments. Short video platforms and short videos have a chance to develop as the Internet revolution continues to intensify and mobile clients gain popularity. This essay examines the challenges involved in producing brief videos that promote a healthy cultural environment in the new context of internet plus, as well as the means of transmitting such videos and creative methods for doing so. Excellent communication content is created in this paper from two perspectives of visual presentation and in-depth meaning, allowing users to fully understand the connotation of a healthy cultural environment. Through the theme of a healthy cultural environment, topic discussion and characteristic activities will be carried out to encourage users' spontaneous sharing of the interactive behavior of communication and the fission communication of brief videos of a healthy environment. This paper develops a model for intelligent recommendation and short video content analysis based on this. In order to further encourage the creative dissemination and development of short videos about healthy cultural environments, the model is used to choose high-quality videos and accurately recommend them to the appropriate users and to serve as an example of how a quick video can be used to communicate innovation and a healthy cultural environment.

## 1. Introduction

The heart and soul of the Chinese people and the source of China's greatest cultural soft power today is the country's excellent and healthy cultural environment. Chinese youth can only fulfil their mission and responsibilities in the new era by bolstering cultural self-confidence, fully reaffirming the value of an excellent, healthy cultural environment, and having absolute faith in its vitality. The gradual development of new media communication forms has opened up new possibilities for the dissemination of a positive cultural environment [1]. Short video is one of the mobile phone clients that is currently undergoing the most rapid development. A short video is one that has a maximum playing time of five minutes. The data from China's research report on network audiovisual development show that people are becoming more and more interested in short videos. One of the key methods for people's daily entertainment and leisure is “brushing” short videos and taking part in creation [2]. Video has gradually evolved into a social “spokesperson” for the dissemination of China's excellent, healthy cultural environment due to its benefits such as fragmentation, scene, portability, and other factors, capturing the interest of a significant portion of the young population. At the same time, the brief video gives more people the opportunity to see Chinese traditional cultural products like Hanfu, calligraphy, Beijing opera, face changing, handicrafts made from bamboo weaving, carpentry, and paper-making [3]. People can better understand the vibrant cultural environment that they have only read about by studying these exquisite craft creations and cutting-edge craft techniques. Short videos used in traditional cultural communication have evolved over time from individualized and entertaining to widespread, organized, and professional. The comments and forwarding volume of short videos about a healthy cultural environment are, however, much lower than their own praise [4] when compared with content about food, beauty, sharing daily life, and other topics. Additionally, users of short videos tend to be young people, while traditional media's audience and market share are gradually declining. This creates a risk to cultural heritage and the marginalization of a vibrant cultural environment. As a result, short video communication channels that promote a healthy cultural environment are proposed.

China has a large number of intangible cultural heritages. Nowadays, many nongenetic inheritors also carry out cultural popularization and dissemination activities on short video platforms, so that more people can know about the life of craftsmen and intangible cultural heritages [5]. Although mobile short video still has some drawbacks, the extensive user base, advanced technical support, high-quality cultural connotation and perfect communication channels together constitute a favorable system to promote the development of traditional culture. The short video mode offers the benefit of channel [6] and is simple to share on mobile media. Short videos are useful for conveying the vibrant traditional culture to viewers while also efficiently exporting the traditional culture to other countries, allowing them to experience and preserve Chinese culture worldwide. Short videos that communicate about Chinese traditional culture are of great quality [7]. The grassroots and young groups of short video platforms compensate for the audience that traditional communication methods have neglected, naturally combine traditional culture with many different types of communication platforms, integrate and innovate traditional culture, realize the benign interaction between them, and provide a sizable audience for the integrated communication of traditional culture. The great traditional culture of China, which serves as the spiritual backbone of the Chinese people, is full of profound philosophical ideas, humanistic ideals, and other admirable traits. These qualities help to mold and promote the Chinese way of thinking and spirituality [8]. The use of brief videos to transmit traditional culture is beneficial for both updating and developing new cultures [9] as well as for the dissemination and selection of Chinese traditional culture.

This paper mainly studies the application of short video in the innovative communication of traditional culture in the new situation of internet plus. Its innovations are as follows: (1) Under the new situation of internet plus, this paper discusses the application of short video in the innovative communication of traditional culture. This paper focuses on constructing the communication mode, communication method, and communication language of traditional culture in mobile short video. The excellent traditional Chinese culture is reshaped and reanalyzed by using the fragmented and fragmented communication mode of mobile short videos. The research of this paper has distinct characteristics of the times. (2) This paper constructs a short video content analysis and intelligent recommendation model and selects high-quality traditional culture short videos from a large number of short videos published by users to share with the corresponding users.

## 2. Related Work

Now, with network technology [10] becoming more and more widespread, it is possible to watch films using mobile clients. Fragmented and low-threshold means of communication are being accepted and used more frequently by people. Short movies are easier to accept and absorb than words and pictures and can give individuals more intuitive knowledge. Short videos are simple to create, disseminate quickly, and are social, and they have quickly emerged as a new driver of Internet industry growth. However, Chinese traditional culture has a rich historical background and is highly valuable for academic inquiry. But studying traditional culture rarely includes looking at the media.

Wan Z argued that traditional culture should innovate its method of transmission by utilizing the popularity of short videos, allowing people to understand traditional culture's significance in addition to its role as a source of entertainment and leisure. This would increase the dissemination of traditional culture and help it leave a more captivating and vivid impression on viewers. Short videos are not only used as a tool in online communities; they are also a platform for users to show off, express their feelings, and share knowledge, according to Santos C et al. [11] They also discussed the adjustment strategies needed for short video content to fit into various community cultures. Caraway B made the point that there are challenges in producing and disseminating short videos, such as challenges with presentation, understanding, and creativity. By employing techniques such modern context adaptation, essence refinement, and spiritual implications, it is vital to maximize distribution [12]. A brief video platform for the incorporation and distribution of traditional Chinese culture was proposed by Ruswandi S. A. in order to encourage the inheritance and development of traditional culture [13, 14]. Dunn et al. summarized and classified the traditional cultural communication content based on mobile short videos and analyzed the short video expressions and picture language with greater influence through the case analysis method [15]. The excellent traditional culture of the nation can be inherited and carried forward [16]. Golding P et al. analyzed the video from the user's visual and auditory perspectives, used multiple DL (deep learning) models to model it, and established multiple DL models to analyze the video in an all-round way [17]. In order to improve the standardization and rigor of the research, Zheng C et al. will use a combination of qualitative and quantitative research methods and pointed out that algorithm recommendation intelligence is one of the important influencing factors [18]. Users' participatory and creative activities in short video apps have a favorable effect on users' perceived value and loyalty, according to Huang J et al. empirical's findings using quantitative analysis techniques [19].

This essay conducts a comprehensive analysis of the use of brief videos in the new context of internet plus for the creative dissemination of traditional culture. This research analyzes and condenses the mobile short movies that showcase traditional culture by looking at the users, platforms, communication contents, communication techniques, forms, and language of mobile short videos. In parallel, a brief movie showcasing traditional culture is proposed as a communication tactic. Based on the foregoing, a model for intelligent recommendation and short video content analysis is created. According to the research, this study has some practical applications and can educate and suggest applications for both traditional cultural innovation communication strategies and short video app recommendation technologies.

## 3. Methodology

### 3.1. Communication Ideas of Traditional Short Cultural Videos

The Chinese nation has a history of thousands of years, and there are countless excellent traditional cultures. At present, most people live in modern metropolises, almost out of touch with traditional culture. With the development and progress of society, the traditional mode of communication is also facing difficulties and problems. With the advent of the new media era, great changes have taken place in the scope, ways, and channels of media communication [20]. In this case, many problems have been exposed in traditional cultural communication, such as the lack of innovation in communication methods, the single subject of communication, and the difficulty in getting the public's approval for the content of communication. Short videos have the characteristics of length and quantity, and people can watch them at any time, regardless of time and place. Video makes use of people's curiosity and demand for information and gradually becomes the main carrier of information. The influx of users has brought business opportunities to the short video platform. This innovation in production and communication brought about by technological development enables traditional culture to be recorded in the original cultural context. At the same time, with the help of short videos, it highlights its artistic charm and expressive tension, thus realizing the modern translation of Chinese excellent traditional culture. The spread of short videos has equal broadcasting rights, and each platform can publish them. Chinese intangible cultural heritage inheritors, craftsmen, and other ordinary people can spread traditional culture through their mobile phones, and the audience can also play short videos at any time. To some extent, this mode of communication has reconstructed the audience of communication culture and added new vitality to the communication of Chinese traditional culture. In 2016, the mobile platform represented by TikTok app was derived, and the beta platform based on live broadcast was gradually popularized among users. Mobile short video platform and live broadcast platform have entered a mature stage.  Figure 1 shows the daily active users in TikTok from 2018 to 2021.

The most common form of communication today is short videos. The advantage of the short video mode is that it is simple to share on mobile media [21]. The dissemination of traditional culture is inextricably linked to contemporary modes of expression, appealing content, and ways of keeping up with trends. Tradition needs to lay down its “Figure” and approach the public's gaze in a more realistic manner. A quick film can encourage the propagation of traditional Chinese culture. The term “activation function” refers to the media's stimulation of material, particularly because users will remark on and forward quick films during transmission, giving the content fresh life, revealing the connection between publishers and audiences, and extending the cultural influence. In order to actualize the visualization and visualization of traditional culture and satisfy the reading habits of users of short video platforms, it is required to adapt the connotation of Chinese traditional culture into an easily understandable video form. The users of short video platforms will be drawn to traditional culture through natural and engaging expressions. In order for consumers to fully comprehend the meaning of traditional culture, the core culture of traditional culture will be uncovered, and good communication content will be created. The audience for mobile short video platforms is categorized by age in Figure 2.

Due to the appearance of short video entertainment software, all social activities of people are entertaining and homogeneous, which is easy for users to have esthetic fatigue. Therefore, it is imperative to spread short videos with cultural connotations. The innovation of traditional culture of short video communication should break through the traditional narrative story mode and show the humanistic feelings in traditional culture. Innovate the expression form of integrated communication of traditional culture, and ensure the diversity of visualization means of Chinese traditional culture. From the aspect of practical creation, how to construct a life-like situational experience needs to apply the research method of semiotics. The recognition of human culture is carried out through symbols. Selecting the cultural symbols of Chinese excellent traditional culture and placing them in short videos will help to shape the life-like situation that conforms to the traditional context. The traditional expression methods of culture need not stick to the inherent forms. When applying short video to cultural communication, diversified forms of expression can make people feel refreshed. At the same time, we can create the cultural brand of traditional culture, introduce users into the next form of cultural communication, promote users to buy products of cultural brands, realize the transformation of economic value, transform the online viewing experience of short videos into offline daily life experience, extend the attitude of traditional cultural communication, and deepen users' experience of traditional culture.

In the short video, the traditional art itself has a multidirectional sensing interaction relationship with the participants and viewers. Through screen-separated interactive behaviors such as display, onlookers, praise, comments, and sharing, all parties make the esthetics complete in the whole-time accompanying social interaction, thus realizing the socialization of the production and dissemination of traditional culture. While creating short videos, the rational use of the original classic works and popular cultural communication programs can undoubtedly effectively improve the efficiency of video output, stimulate people's interest, and guide people to watch the full version of videos, which can make the transmission of traditional culture more efficient. In view of the traditional culture with complex content, the length of short video cannot present all the content, but it can adopt the classical lens to provide detailed information about the traditional culture. Because traditional culture has more IP, it can be developed around animation, variety shows, games, movies, and other forms. Traditional culture can use short video to spread, reduce the distance between audience and traditional culture, and use high technology to reduce users' sense of screen distance, so that users and traditional culture have a sense of closeness. In addition, short video works should not only find another way to express content, voice style, narrative perspective, and breakthrough point, but also work hard on cultural connotation and ideological guidance.

### 3.2. Short Video Content Analysis and Intelligent Recommendation

In order to improve recollection rates and decrease manslaughter rates, this research develops a DL model to swap out the original standard machine learning model [22]. By introducing multiple hidden layers, DL first extracts the low-level features of the data to be measured and then combines the low-level features in a linear or nonlinear way to form more abstract high-level features from shallow to deep, achieving a deep nonlinear network structure, representing the input data, realizing complex function approximation, and showing a powerful ability to learn the key features of data sets from a few sample sets.  Figure 3 displays the DL model.

Recommendation system architecture is usually divided into content modeling layer, interest modeling layer, and user interaction layer. In the content modeling layer, the structure of short videos is analyzed mainly by analysis tools. The user interaction layer records the behavior information related to users, classifies users, and constantly updates the basic attributes of users. The interest modeling layer is the core link. After the interaction between semantic analysis layer and user interaction layer, the user's portrait on the platform will be gradually generated. The machine learning algorithm will train the user's interest model, improve the accuracy of model matching, and complete high-quality algorithm recommendation. The algorithm architecture design process is shown in Figure 4.

Better communication results can be produced for less money if the video content is of a good caliber and the platform's recommendation process is used responsibly. The phenomena of erroneous content suggestion and unsystematic recommendation stream information readily happen in the process of cold start in the interaction between users and short video app, which impacts users' content appraisal of the platform. Monitoring the information that is presented by search results is more effective than tracking users' long-term preferences, and even some users' “temporary thoughts” can be identified. It is crucial to suitably incorporate some manual tasks into the recommendation of short videos in addition to letting intelligent algorithms entirely dominate the distribution of short videos. The formula gives the following description of the reset's residual learning module:

(1) $$\begin{array}{c} y=F\left(x,\left\{\text{Wi}\right\}\right)+x. \end{array}$$

For the input *x*, parameter learning is performed through the intermediate function *F*(*x*, *w*), and *F* is what we call the residual function. Two gated states are obtained through the last transmitted state *h*^*t*−1^ and the input *x*^*t*^ of the current node. Among them, *r* controls the gate of reset, and *z* is the gate of control update and is calculated as follows:

(2) $$\begin{array}{c} r_{t}=\text{Sigmoid}\left(W_{r}\cdot \left[h_{t-1},x_{t}\right]\right),\\ z_{t}=\text{Sigmoid}\left(W_{z}\cdot \left[h_{t-1},x_{t}\right]\right). \end{array}$$

Calculate the candidate hidden layer ${\tilde{h}}_{t}$, which represents the new information at the current moment, where *r*_*t*_ is used to control how much previous memory needs to be retained. The information calculation formula of the current word is as follows:

(3) $$\begin{array}{c} {\tilde{h}}_{t}=\text{Tanh}\left(W\cdot \left[r_{t}*h_{t-1},x_{t}\right]\right). \end{array}$$

Finally, *z*_*t*_ controls how much information needs to be forgotten from the hidden layer *h*_*t*−1_ at the previous moment, and how much information ${\tilde{h}}_{t}$ of the hidden layer at the current moment needs to be added. Finally, *h*_*t*_ is obtained, and the hidden layer information of the final output is directly obtained. The calculation formula is as follows:

(4) $$\begin{array}{c} h_{t}=\left(1-z_{t}\right)*h_{t-1}+z_{t}*{\tilde{h}}_{t}. \end{array}$$

Given the input gate activation value *i*_*t*_, the forget gate activation value *f*_*t*_, and the candidate state value *C*, calculate the new state *t* of the *C*_*t*_ storage unit in time:

(5) $$\begin{array}{c} C_{t}=i_{t}*{\tilde{C}}_{t}+f_{t}*C_{t-1}. \end{array}$$

With the new state of the memory cell, we can calculate its output gate activation value and then its output value:

(6) $$\begin{array}{c} O_{t}=\sigma \left(W_{o}x_{t}+U_{o}h_{t-1}+V_{o}C_{t}+b_{o}\right). \end{array}$$

The verification set and training set mean files are produced. It is equivalent to the process of feature vector normalization after the mean value has been removed from the image. The training effect is better, and the accuracy rate is higher with more regular data than with less regular data. To get the mean, one must average all training sample data. Once calculated, save it as a mean file so that you can use it to subtract without having to recalculate the test images. In order to gather customer input, many video websites have options for either satisfactory or unsatisfactory ratings. The suggested algorithm technology must be in constant communication with the user's usage patterns in order to update and improve performance. As a result, evaluating the empirical outcomes of intelligent algorithm recommendation from the perspective of the user might offer a fresh approach for enhancing the technological model. Assumption:

(7) $$\begin{array}{c} \text{Userproflie}\left(c\right)=\left(w_{c1},w_{c2},\cdots ,w_{\text{ck}}\right), \end{array}$$

where *w*_*ci*_ represents the importance of keyword *k*_*i*_ to user *c*. Content(*s*) represents the content characteristics of video *s*, that is, the set of phrases that describe the characteristics of video *s*. I have added it in the corresponding place. Then, in the content-based recommendation, user *c*'s preference score *r*_*cs*_ for video *s* is defined as

(8) $$\begin{array}{c} r_{\text{cs}}=\text{Score}\left(\text{Userproflie}\left(c\right),\text{Content}\left(s\right)\right). \end{array}$$

There are different methods to calculate score, for example, the distance calculation method of cosine of vector included angle in the simplest information retrieval field can be used:

(9) $$\begin{array}{c} r_{\text{cs}}=\text{Cos}\left({\overset{⟶}{w}}_{c},{\overset{⟶}{w}}_{s}\right)=\frac{\sum_{i=1}^{k}w_{\text{ic}}w_{\text{is}}}{\left(\sqrt{\sum_{i=1}^{k}{w^{2}}_{\text{ic}}}\sqrt{\sum_{i=1}^{k}{w^{2}}_{\text{is}}}\right)}. \end{array}$$

Finally, objects such as text can be sorted according to the obtained *r* value, and videos can be recommended to users.

The platform can promote the operation of the whole recommendation system through the combination of intelligent distribution and fan distribution and achieve more accurate recommendation firmly around user preferences. Therefore, the content that users brush is a comprehensive recommendation based on algorithm attribute + real-time popularity + user relationship, which can effectively prevent users from falling into information cocoon room, and operation is an invisible hand behind it. The algorithm recommendation of the platform is accurate enough, and users will naturally like the pushed content in the process of using it, giving it a high evaluation, so as to promote the innovation and dissemination of traditional culture.

## 4. Result Analysis and Discussion

This chapter's model construction was simulated. The Internet-based questionnaire platform is the primary method used by the algorithm intelligent scale to gather data, and the network channel is the primary method used to distribute the questionnaire. This study first checked the accuracy of the data in order to confirm the quality of the initial questionnaire. The results of the validity and reliability tests for the intelligent scale for algorithm recommendation are shown in Table 1.

From Cronbach *α* coefficient analysis, it can be seen that the reliability coefficient of intelligent algorithm recommendation reaches 0.931. Through KMO value analysis, we can know that in the validity test of intelligent scale for algorithm recommendation, KMO value reaches 0.894, which is higher than 0.6 required by quality. Moreover, the mean file in your own field is different from the mean file on Imagenet. During the experiment, the data set is divided into training set and testing set. The algorithm works in the training set and predicts the items in the testing set through the data in the training set. In caffe, tensorflow environment without GPU version, there is a high requirement for training time. This paper hopes that the training can be completed in the shortest possible time. Whether it is the training of avatar images on caffe or the training on tensorflow after video frame extraction, it is hoped that the classification training can be completed within 2 hours.  Figure 5 shows the intelligent gravel map recommended by the algorithm.

According to the feedback result of gravel map, this algorithm recommends intelligent exploratory factor analysis to precipitate four factors, and the factor loads of each factor's measurement items are all greater than 0.5, and there is no obvious cross load phenomenon. Comparison of recall results of different algorithms is shown in Figure 6.

Accuracy aims to measure whether an algorithm recommendation system can push content products that meet users' preferences. This kind of label is usually explicit and can quickly capture information, such as the user's place of residence, gender, and attention to users. The qualified algorithm recommendation should acquire and form the user's interest model, and be able to get personal tags according to the user's attribute analysis, which can match the user's interests and attributes and meet the most basic personalized recommendation. Comparison of accuracy results of different algorithms is shown in Figure 7.

The validation sample set and training set are extracted, and the val samples with a set ratio are randomly obtained from the set rawdata folder, and the rest are train samples. The ratio of positive and negative samples in this project is initially set at 3 : 7. Because the positive and negative samples need to be balanced, when the positive and negative samples are extremely unbalanced, the characteristics of the side with fewer samples will be weakened by the side with stronger samples. The intelligent confirmatory factor analysis of the recommended algorithm is shown in Table 2.

Through the model fitting of intelligent latent variables recommended by the algorithm, the index of model fitting degree is up to standard. Generally speaking, the intelligent model fitting degree recommended by the algorithm is at an acceptable level. The experimental results in this chapter show that the recall rate of this algorithm can reach 94.12%, which is 9.31% higher than the traditional collaborative filtering method. At the same time, the algorithm in this paper has high accuracy and certain reliability.

## 5. Conclusions

Everyone can publish short videos in the modern, sophisticated world. The process of brief video transmission can be completed by the audience watching, commenting, and forwarding as long as individuals continue to collect, record, edit, and distribute videos using mobile devices. The qualities and communication benefits of mobile short video platforms are examined in this study, along with the concepts, psychology, and characteristics of the users using the theories of communication, sociology, and psychology. At the same time, it examines the mobile short video-based traditional culture communication strategy in an effort to merge traditional culture with network growth in order to transmit it rapidly and effectively. It is possible to improve communication outcomes while spending less money if the video content is of a good quality and the platform's recommendation function is used responsibly. A model for intelligent recommendation and short video content analysis is created using this information. According to experimental findings, this algorithm may achieve a recall rate of 94.12%, which is 9.31% higher than the typical collaborative filtering approach. This algorithm also has a high level of accuracy. The application of short video app recommendation technology and the communication strategy of traditional culture innovation can both benefit from this research's practical value, which can offer guidance and suggestions. Knowing the traits of production communication is crucial for innovating production communication routes and promoting high-quality traditional culture to users. At the same time, we should encourage the spread of a brief video showcasing excellent Chinese traditional culture to various service industries and supporting industries in order to continuously create new conditions for its growth. The work done in this paper is extremely limited, and the proposed algorithm also has some drawbacks as a result of time and technological constraints. Although this research still has certain issues, these will be fixed in the future.

## Figures and Tables

**Figure 1:** Daily active users in TikTok from 2018 to 2021.

**Figure 2:** Age distribution of audience of mobile short video platform.

**Figure 3:** DL model.

**Figure 4:** Flow chart of algorithm architecture design.

**Figure 5:** Algorithm recommends intelligent gravel map.

**Figure 6:** Recall results of different algorithms.

**Figure 7:** Accuracy results of different algorithms.

**Table 1:** Reliability and validity test results of algorithm recommendation intelligent scale.

Name	CITC	Term removed *α* coefficient	Cronbach *α* coefficient	KMO
RS1	0.718	0.948	0.931	0.894
RS2	0.706	0.948	—	—
RS3	0.668	0.948	—	—
RS4	0.620	0.951	—	—
RS5	0.715	0.948	—	—
RS6	0.702	0.948	—	—
RS7	0.718	0.948	—	—
RS8	0.637	0.951	—	—
RS9	0.675	0.948	—	—
RS10	0.686	0.948	—	—
RS11	0.639	0.951	—	—
RS12	0.664	0.951	—	—
RS13	0.525	0.952	—	—
RS14	0.605	0.951	—	—
RS15	0.646	0.951	—	—
RS16	0.734	0.950	—	—
RS17	0.786	0.949	—	—
RS18	0.775	0.949	—	—
RS19	0.764	0.949	—	—
RS20	0.768	0.949	—	—

**Table 2:** Intelligent confirmatory factor analysis for algorithm recommendation.

Accuracy	RS1	0.87	Novelty	RS11	0.79
	RS2	0.86		RS12	0.81
	RS3	0.84		RS13	0.59
	RS4	0.70		RS14	0.70
	RS5	0.76		RS15	0.82

Diversity	RS6	0.81	Surprise	RS16	0.84
	RS7	1.84		RS17	0.86
	RS8	0.70		RS18	0.85
	RS9	0.81		RS19	0.85
	RS10	0.80		RS20	0.83

## Data Availability

The data used to support the findings of this study are available from the corresponding author upon request.
